The article "Glycinebetaine mitigates drought stress-induced oxidative damage in pears" was retracted in 2022. Reasons: compromised peer review; a conflict of interest; concerns about the authorship.

# Glycinebetaine mitigates drought stress-induced oxidative damage in pears

**DOI:** 10.1371/journal.pone.0251389

**Published:** 2021-11-18

**Authors:** Tiequan Niu, Tianpeng Zhang, Yue Qiao, Pengfei Wen, Guangqian Zhai, Enke Liu, Dhafer A. Al-Bakre, Mohammad S. Al-Harbi, Xiuping Gao, Xinghong Yang

**Affiliations:** 1 College of Horticulture, Shanxi Agricultural University, Taigu, China; 2 College of Life Science, Shandong Agricultural University, Taian, China; 3 Institute of Agricultural Resources & Economy, Shanxi Academy of Agricultural Sciences, Taiyuan, China; 4 Shanxi Province Key Laboratory of Organic Dry Farming, Arid Farming Research Center, Shanxi Academy of Agricultural Sciences, Taiyuan, China; 5 Department of Biology, College of Science, University of Tabuk, Tabuk, Saudi Arabia; 6 Department of Biology, College of Science, Taif University, Taif, Saudi Arabia; 7 Key Laboratory of Crop Gene Resources and Germplasm Enhancement on Loess Plateau, Ministry of Agriculture, P. R. China, Taiyuan, China; Harran Üniversitesi: Harran Universitesi, TURKEY

## Abstract

Glycinebetaine (GB) is an osmoprotectant found in plants under environmental stresses that incorporates drought and is associated with drought tolerance in several plants, such as the woody pear. However, how GB improves drought tolerance in pears remains unclear. In the current study, we explored the mechanism by which GB enhances drought tolerance of whole pear plants (*Pyrus bretschneideri* Redh. cv. Suli) supplied with exogenous GB. The results showed that on the sixth day after withholding water, levels of O_2_·^−^, H_2_O_2_, malonaldehyde (MDA) and electrolyte leakage in the leaves were substantially increased by 143%, 38%, 134% and 155%, respectively. Exogenous GB treatment was substantially reduced O_2_·^−^, H_2_O_2_, MDA and electrolyte leakage (38%, 24%, 38% and 36%, respectively) in drought-stressed leaves. Furthermore, exogenous GB induced considerably higher antioxidant enzyme activity in dry-stressed leaves than drought-stressed treatment alone on the sixth day after withholding water, such as superoxide dismutase (SOD) (201%) and peroxidase (POD) (127%). In addition, these GB-induced phenomena led to increased endogenous GB levels in the leaves of the GB 100 + drought and GB 500 + drought treatment groups by 30% and 78%, respectively, compared to drought treatment alone. The findings obtained were confirmed by the results of the disconnected leaf tests, in which GB contributed to a substantial increase in SOD activity and parallel dose- and time-based decreases in MDA levels. These results demonstrate that GB-conferred drought resistance in pears may be due in part to minimizing symptoms of oxidative harm incurred in response to drought by the activities of antioxidants and by reducing the build-up of ROS and lipid peroxidation.

## Introduction

Drought stress is one of the most serious abiotic stresses limiting plant growth, development, health and productivity [1–3]. Drought stress can trigger several responses in plants, including reducing the growth of shoots, inhibiting the initiation of new leaves and accelerating the senescence of old leaves, leading to decreased biomass production and yield [4–7].

Plants react by modifying cellular metabolism and triggering defensive mechanisms to adjust to drought stress [8]. Oxidative bursts can be found in plants’ reactions to drought stress [9, 10]. Such activity is attributed to an imbalance in the development and scavenging of reactive oxygen species (ROS), such as radicals for superoxide anions (O_2_·^−^), hydrogen peroxide (H_2_O_2_), and hydroxyl radicals (OH). ROS regularly induce metabolic processes, including breathing, photosynthesis, lignification and aging, adequately controlling the equilibrium between development and quenching. Imbalanced mechanisms can inflict oxidative harm to plants triggered by stress [11]. Accumulating data have shown that drought stress contributes to ROS surplus in plant development [12, 13]. Excessive ROS levels are incredibly toxic and can cause dramatic effects on plant cells through lipid peroxidation, protein degradation and DNA fragmentation, inevitably leading to cell death [14–16].

Plants naturally employ defense processes, such as superoxide dismutase (SODs), catalase (CAT) and peroxidase (PODs), and nonenzymatic antioxidants, such as glutathione and ascorbic acid, to counteract the cytotoxic effects of ROS through antioxidant systems [17–19]. These nonenzymatic and enzymatic antioxidants play a key role in guarding against the abiotic stresses of overproduced ROS [20]. SOD is a family of metalloenzymes used in the production of H_2_O_2_ and oxygen in scavenging O_2_·^−^ that plays an important role in cellular defense against cytotoxic superoxide radicals. In addition to SOD, other enzymes, the most important being CAT and PODs, regulate the intracellular H2O2 levels. CAT diverts H_2_O_2_ into water and oxygen, while POD reduces H_2_O_2_, which is used as an electron donor substrate, into water [21].

The aggregation of osmolytes in cells, such as glycinebetaine (GB), typically responds to numerous environmental pressures, including drought, salinity and extreme temperature [22–26]. GB, one of the most prevalent and powerful osmoprotectants in a number of higher plants, is an environmentally healthy, nontoxic and water-resoluble osmolyte [27–34]. Resistance to stress due to various abiotic pressures has been recorded to be associated with GB accumulation [35–48]. GB also protects plants through the stabilization of membranes, proteins and enzymes in addition to its function as an osmoprotectant [28, 49–51]. In addition, where transformed genes are overexpressed for GB synthesis, plants exhibit improved drought resistance [31]. It has been suggested that exogenous GB application enhances resistance to drought in many plants by preventing photoinhibition [52] or by upregulating antioxidant enzymes [29, 35, 36, 53, 54].

Our previous study showed that accumulation of water stress-induced GB is correlated with pear drought resistance [36]. However, to date it is uncertain how GB alleviates drought-induced oxidative stress, increases poultry resistance and protects poultry plants from oxidation. In this research, exogenously administered GB protected plants against oxidative drought, which was correlated with increased endogenous GB aggregation in pears, via inhibition of ROS formation, decreased lipid peroxidation and increased enzymatic antioxidant capacities. To our knowledge, this is the first study examining the efficacy of GB in reducing oxidative stress in a woody plant under drought stress.

## Materials and methods

### Plants and test design

Two sets of tests were performed by the researchers: one using entire pear plants and the other on single leaves, which are referred to as whole plant evaluation and isolated leaf trial, respectively.

### Experiments on both species

Experiments on "Birchleaf pear" (*Pyrus betulaefolia* Rehd.) were performed in a greenhouse with the use of 2-year-old ’Suly’ pear trees grown in pots with a diameter of 45 cm and a depth of 35 cm, and every pot was completed with 25 kg of the topsoil/river sand/decomposed sheep manure mixture and 3:1:1 and 1 kg m^−3^ superphosphate. Prior to care, plants with comparable vigor for development were picked and watered equally well. The withholding of water was used to simulate drought. Pear plants were handled with 100 or 500-mg foliar sprays L^−1^ GB with 0.02% Tween 20 (v/v) ("GB 100 + drought") and "GB 500 + drought" therapies, on the day that the water was withheld, and 0.02% Tween 20 (v/v) of the same amount of water was sprayed onto the control unit feed ("Drought" treatment). The other experiment involved the handling of well-watered plants with a comparable amount of 0.02% Tween 20 (v/v) water spraying, but these plants were well watered throughout the entire trial ("well-watered" treatment). The plot architecture was a total randomized block of six single tree replications.

Five mature leaves were collected between 16:30 and 17:30 from the center of each plant’s crop at various time intervals 0, 3 and 6 d after spraying. After removal of the central veins, the leaf sample was instantly ground into powder using liquid N_2_ that was primed for immediate application or deposited at -80°C for further study. On the same day, the weight and pressure chamber system were used to calculate the soil water content and leaf water capacity based on the method mentioned above in Gao, Pan [55] to provide a true approximation of the amount of water stress. Soil samples were obtained by a bore from a certain position in each container, which spanned deep to the bottom of the pot, before 10:30 am. At approximately 6:30 am, the leaf water capacity was assessed immediately after the removal of leaves from the shoots.

### Experiments on detached leaves

The mature leaves of "Suly" (*Pyrus bretschneideri* Rehd.) trees greased on the "Birchleaf" (*Pyrus betulaefoli*) rootstocks grown open-field were removed from the center of the strongly grown footsteps of approximately 12-year-old "Suly." Two separate leaf studies were undertaken. In the first experiment, we studied the impact on SOD behavior and MDA content in response to varying concentrations of GB in separate pear leaves during the process of water loss. At approximately 8:30 and 9:30 am, the leaves were sampled and processed immediately. Ten leaves were randomly picked for each treatment. Immediately after collection, a group of 10 leaves that were neither dehydrated nor GB-treated were frozen in liquid N_2_ for monitoring. For the other leaves, solutions of various amounts of GB treatment (50, 100, 500, 1,000 and 5000 mg L^−1^) were measured, and the solution was allowed to penetrate under vacuum for 10 min. Another process involved infiltration of bottled water in the leaves. The leaves were dried by air after infiltration and placed on a yarn grid. As the water loss approached the initial fresh weight, the leaves were ground into a fine powder with liquid N_2_ and processed at –80°C until further examination.

We analyzed the duration of improvements in SOD and MDA quality in different pericarbons following GB treatment in the second experiment. As in the aforementioned experiment, leaf samples were gathered and then altered into two classes. One of the leaves was vacuumed for 10 min and weighed after exposure to 500 mg L^–1^ GB solution. The leaves were loaded into a net and weighed 0, 30, 60, 90, 120, 180 and 240 min after infiltration. Then, they were ground into a fine powder with liquid N_2_ and stored at f ‐80°C for further study. The other leaves were washed with purified water in the same way.

### GB quantification and extraction

Essentially, we adopted the Rhodes, Rich [56] alteration of the protocol. A ceramic mortar comprising 2 ml methanol, chloroform and 0.2 M KHCO_3_ (12/5/1, v/v/v) mixture was used to grind leaf samples (500 mg). For 30 min, the blended liquid was incubated in a water bath at 60°C and was then centrifuged at 10,000 livres for 10 min. The aqueous process was separated by amberlite CG-50 and Dowex 1-X2 ion-exchange resins. NH_4_OH (4 M) was eluted and dried on a 57°C stream spinning evaporator. The chosen sample was dissolved in 2 mL of methanol for chromatography. A liquid column (SCL-10AVP; Shimadzu, Kyoto, Japan), fitted with a Hypersil SCX column, was used to examine the distilled extract comprising GB.

### Enzyme extraction and assays

Frozen leaf samples (0.5 g) were placed into jars with 5 mL of cold mining buffer consisting of 50 mM potassium (pH 7.0), 1 mM EDTA and 5% (w/v) polyvinylpolypyrrolidone (PVPP). Furthermore, samples were ground into a fine power by means of liquid N_2_. The powder was homogenized at 15,000 g/min at 4°C and then centrifuged for 20 min. The supernatant was used for the enzyme and complete protein tests described below according to a process already defined by Giannopolitis and Ries [57]. SOD (EC 1.15.1.1) activity was measured by NBT (nitro blue tetrazolium) photochemical reduction inhibition. The 3 mL reaction mixture comprised 50 mM potassium phosphate buffer (pH 7.8), 13 mM methionine, 2 mm riboflavin, 0.1 mM EDTA, 75 mM NBT, and 100 μL of enzyme extract. The mixture was illuminated for 15 min at 5,000 lx. In addition, the amount of enzyme needed to cause a 50% inhibition of NBT as monitored at 560 nm was specified as a unit of SOD activity. SOD activity is expressed as U mg^−1^ protein.

After ingestion of H_2_O_2_ (extinction core 39.4 mM^−1^ cm^−1^) at 240 nm for three min [58], the behavior of CAT (EC 1.11.1.6) was calculated. The reaction mixture contained 2.5 mL in 50 mM PTS (pH 7.0), 300 μL in 15 mM H_2_O_2_, and 200 μL in the enzyme extract. The function of the enzyme is expressed as the mg^−1^ protein min^−1^ decreased by μmol H_2_O_2_.

The POD (EC 1.11.1.7) activity was identified in guaiacol oxidation reactions as previously defined by Chance and Maehly [59] at 470 nm for 3 min (extinction coefficient 26.6 mM^−1^ cm^−1^). The 3-mL mixture included 1 mL potassium phosphate buffer (pH 7.0), 1 mL guaiacol 1%, 0.9 mL of 0.2 M H_2_O_2_ and 100 μL enzyme extract. Enzyme extract was used for a 1 mL reaction. The activity of μmol mg^−1^ protein min^−1^ is expressed as POD.

### Protein determination

A method previously described in Bradford [60] with standard BSA was used to calculate protein concentration.

### H_2_O_2_ calculation

H_2_O_2_ was evaluated with a minor adjustment in conjunction with the procedure already defined by Alexieva, Sergiev [61]. The batch of frozen leaves (0.5 g) was further ground into a fine powder using liquid N_2_ and homogenized in 5 mL of 3% trichloroacetic acid (TCA) with 10 mM EDTA in an ice bath. The homogenate was centrifuged at 15,000 ×g for 15 min. Then, 0.5 mL of supernatant was mixed with 0.5 mL, 10 mM (pH-7.0) and 1 mL of 1 mM potassium iodide (10 mM) in potassium phosphate buffer. The reaction was then performed in the dark for 1 h, and the absorbance was read at 390 nm. H_2_O_2_ was determined based upon a regular H_2_O_2_ curve and is expressed as fresh weight of μmol g^−1^.

### Measurement of O_2_·^−^

The O_2_·^−^ content was measured in conjunction with the Elstner [62] method mentioned above. The tracking of nitrite formation in the presence of O_2_·^−^ from hydroxylamine at 530 nm absorption was calculated.

### Lipid peroxidation

Lipid peroxidation was estimated following the process previously defined by Heath and Packer [63] with minor changes using the calculation of the sum of malondialdehyde (MDA) as a final product of lipid peroxidation. Leaf samples (0.5 g) were ground with liquid N_2_ into a thin powder, which were then mixed with 5 mL of 5% (w/v) TCA and homogenized. The homogenates were combined with 4 mL thiobarbituric acid (TBA; 0.6% TBA in 20% TCA) at 12,000 ×g for 15 min. The reaction mixture was heated for 30 min in a water bath at 95°C, cooled down rapidly in an ice bath and then centrifuged for 15 min at 12,000 ×g. Absorbance of the supernatant was estimated at 532 nm by eliminating absorption at 600 nm and 450 nm for nonspecific turbidities. MDA concentration was determined using the following formula from the absorption gap at 532, 600 and 450 nm:

MDA = 6.45 (A_532_ − A_600_) - 0.56 A_450_

Nmol g^−1^ FW represents MDA concentration.

### Leakage in electrolytes

Due to the technique previously mentioned by Valentovic, Luxova [64], electrolyte leakage (EL) was used to evaluate membrane permeability with limited modifications. Ten disks (5 mm diameter) were washed with water, placed in shut vials containing 20 ml distilled water and incubated for 24 hours at room temperature. Electrical solution conductivity (L1) was developed. Samples were autoclaved to a temperature of 120°C for approximately 20 min to release all electrolytes, and the final electrical conductance (L2) was calculated. EL (%) = (L1/L2) = equivalent to 100 was calculated.

### Statistical analysis

Data were preprocessed using SigmaPlot 12.0 (Systat Software, Erkrath, Germany), and pre-existing data were produced through Microsoft Excel 2010 (Microsoft, Redmond, WA). The study of variation using SAS software (SAS 8.1 version; SAS Institute, Cary, NC) and Student’s t-test at *P* < 0.05 (*) and *P* < 0.01 (**) was used to evaluate significant variations between data. At least three replicates of data are shown as average values ± SD.

## Results

### The effects GB application on the production of O_2_·^−^ and H_2_O_2_ in plant leaves stressed by drought

ROS development, particularly O_2_·^−^ and H_2_O_2_, is an increasingly recognized response to environmental stresses from almost all plant species when they are exposed to dry pressure [65]. In this analysis, levels of O_2_·^−^ and H_2_O_2_ in the leaves of pear plants were examined under conditions of drought stress. The day that water was withheld, 100 or 500 mg L^−1^ GB was sprayed onto the leaves of potted pear seedlings. When plants were subjected to mild and moderate drought stress on the third and sixth days after water withdrawal (GB spraying), respectively, O_2_·^−^ in the leaves of the sewer-treated plants without GB treatment significantly increased their production (40% and 143%, respectively) relative to water-resistant controls (Fig 1A). Increased production of O_2_·^−^ in dry-stressed blooms, which occurred in a dose- and time-dependent manner (Fig 1A), was significantly inhibited by GB foliar application. Treatment with 500 mg L^−1^ GB decreased drought-induced stress-induced O_2_·^−^ production by 21% and 38% on the third and sixth days, respectively, after GB application.

**Fig 1:** Impact of glycinebetaine (GB) spray application on levels of O_2_·^−^ (A) and H_2_O_2_ (B) in the blood of pear planting under drought-related stress conditions. On the day of water preservation, the foliage of pear plants was sprayed with a GB solution of 0 (Drought), 100 (GB 100 + drought) or 500 mg L^−1^ (GB 500 + Drought). The same volume of water was added to well-watered plants. On the third and sixth days of the GB foliar spray (or water retention), soil water levels and leaf water capacity culminated in both the "dryness" and the "GB + drought" classes undergoing mild and severe drought tension. Asterisks demonstrate considerable variations from watery plants (* *P* < 0.05, ** *P* < 0.01, Student′s *t*-test). Six replicates are shown as the mean ± SD.

Likewise, the development of H_2_O_2_, which was similar to the production of O_2_·^−,^ displayed a response trend to drought stress and GB application (Fig 1A and 1B). Drought stress also dramatically improved H_2_O_2_ development (38%) to a degree greater than the well-watered regulation within 6 d of stress treatment (Fig 1B). Dose- and time-dependent usage of foliar GB greatly decreased the amount of H_2_O_2_ in dry-stressed leaves (Fig 1B). H_2_O_2_ levels in the leaves of the GB 500 + dryness group were significantly reduced to a low level (24%) on the sixth day after GB application compared to levels in drought alone leaves (Fig 1B).

### The effects of GB application in the leaves of dried plants with lipid peroxidation and membrane degradation

Overproduction of ROS may cause cell membranes to undergo lipid peroxidation. MDA content is often used as an index of lipid peroxidation and was measured in dry plants in this study. As shown in Fig 2, the leaves of basic drought-treated plants induced a substantial improvement in MDA (38% and 134%) compared to the well-watered controls on the third and sixth days after water was maintained (Fig 2A). Drought-induced MDA output drastically decreased with GB implementation (Fig 2A). When plants experienced moderate drought stress (Table 1), MDA levels increased in the leaves of single plant dryness treated on the third day after application of GB (withholding of water), and only small shifts in MDA concentrations were observed in the leaves of the GB (100 or 500 mg L^–1^) plus dryness treatment classes (Fig 2A). Levels of MDA were considerably lower in GB leaves (100 or 500 mg L^‐1^) on the sixth day following GB application when the plants were subjected to moderate drought stress (Table 1) compared to simple, drought-treated plants (Fig 2A).

**Fig 2:** Glycinebetaine (GB) foliar pellet effects in the leaves of pear seedlings under drought stress (MDA material (A) and electrolyte leakage (B)). The foliage was sprayed on the pear plants with GB solution of 0 (Drought), 100 (GB 100 + drought) or 500 mg L^−1^ (GB 500 + drought). Well-watered plants with the same amount of water were also sprayed. Depending on the content of soil water and the water capacity, on the third and sixth days after foliar spraying (or withholding of the water), both the "Drought" and "GB + dryness" classes exhibited mild and severe drought stress characteristics. Important discrepancies are shown between asterisks and well-watered plants (* *P* < 0.05, ** *P* < 0.01, Student′s *t*-test). Six replicates of the data are shown as the mean ± SD.

**Table 1:** Evaluation of plant water status during the experimental period.

Days after withholding water	Treatment	Soil water content (%)	Leaf water potential (MPa)	Evaluated plant water status
0	Well-watered	24.8	−0.41	No stress
	Drought	25.0	−0.40	No stress
	GB 100 + Drought	24.8	−0.41	No stress
	GB 500 + Drought	24.9	−0.41	No stress
3	Well-watered	24.8	−0.41	No stress
	Drought	13.6**	−0.66**	Mild drought
	GB 100 + Drought	14.1**	−0.63**	Mild drought
	GB 500 + Drought	13.8**	−0.64**	Mild drought
6	Well-watered	25.0	−0.40	No stress
	Drought	9.0**	−0.90**	Moderate drought
	GB 100 + Drought	9.3**	−0.83**	Moderate drought
	GB 500 + Drought	9.5**	−0.78**	Moderate drought

Asterisks indicate significant differences compared to well-watered plants (** *P* < 0.01, Student′s *t*-test).

We next examined the EL of pear plants to further assess the impact of drought stress on membrane injury. Cell membranes of drought-stressed blades were also degraded due to drought stress, which corresponded to increased EL levels (Fig 2B). Drought stress-induced membrane degradation, however, was substantially alleviated by GB application, depending on the dose and time (Fig 2B). Compared to the well-watered controls, on the third day after water retention (Application GB), EL increased by 19% in the florets of drying-treated plants without GB treatment, but application of 100 or 500 mg GB on drought-stressed EL almost entirely arrested this process (Fig 2B). On the sixth day after application, EL was increased by 155% in plants alone, which was higher than the well-watered plants, in the leaves of plants that had been subject to dryness care, whereas the GB application was slightly reduced at 100 or 500 mg L^−1^ relative to plant leaves subject to dry weight stress (23% and 36%, respectively).

### Effects of GB application on the antioxidant activity of plant leaves stressed by drought

Plants have different methods for avoiding oxidative harm by triggering their antioxidant protection mechanisms. In these strategies, various antioxidant enzymes, such as SOD, POD and CAT, play an important role [66]. Our findings showed that application of GB to the leaves of pear plants experiencing dryness also increased the activity of SOD, POD, and CAT (Fig 3A–3C). Under dry stress conditions, the simple plants treated with drought exhibited considerably higher SOD activity than well-watered controls (Fig 3A). Use of GB further improved the dose- and time-dependent dry stress-reducing SOD activity in plants (Fig 3A). On the sixth day following GB application, when plants were under moderate drought stress (Table 1), in the leaves of basic, well-watered plants, SOD activity increased by 122%, and we found that there was even higher (201%) SOD activity in the GB 500 + drought treatment group, illustrating significantly increased SOD activity in the leaves.

**Fig 3:** Effects of the application of glycinebetaine (GB) to the leaves of pear seedlings under drought stress for SOD (A), POD (B) and CAT (C). The foliage was sprayed on pear plants with GB solution of 0 (Drought), 100 (GB 100 + drought) or 500 mg L^−1^ (GB 500 + drought). Well-watered plants with the same volume of water were also sprayed. On the third and sixth days of GB foliar spray (or water retention), soil water levels and leaf water capacity culminated in both the "dryness" and the "GB + drought" classes undergoing mild and severe drought tension. Important discrepancies are shown by asterisks compared to well-watered plants (* *P* < 0.05, ** *P* < 0.01, Student′s *t*-test). Six replicates of the data are shown as the mean ± SD.

Likewise, in contrast to the well-watered management of basic drought-treated plants, drought stress dramatically improved POD activity within 6 ds of the water retained (Fig 3B). The use of GB increased the dose- and time-dependent dry stress-induced POD activity in plants (Fig 3B). On the sixth day following application of GB, POD activities in the simple dry-treated leaves were considerably higher (68%) than those in the well-watered control; nevertheless, in leaves of the GB 500 + drought treatment group, we observed even higher (127%) POD activity (Fig 3B). During drought stress, CAT activity in the simple plant leaves improved slightly to a degree higher than that under well-watered regulation; however, CAT activity in the GB 500 + drought treatment community was slightly higher than that above, while it varied insignificantly from that under simple dry-treated plant activity (Fig 3C).

### Effects of GB application on endogenous GB accumulation in the leaves of drought-stressed plants

Exogenous GB treatment can help mitigate adverse environmental stress effects and boost the degree of endogenous GB [31, 44, 54, 66–68]. In this study, the day the water was withheld, GB was sprayed onto potted pear seedlings at 100 or 500 mg L^−1^. On the third day after spraying, when the plants were exposed to mild drought stress, endogenous GB levels in the leaves of simple plants treated with drought were substantially increased (32% and 91%, respectively), and in the leaves of the GB 100+Drought and GB 500+Drought treatment groups, we observed higher levels of endogenous GB than in the leaves of plants subjected to drought alone. On the 6th day of spraying, endogenous GB (30% and 78%, respectively) of both treatment classes was already higher than that of plant leaves subjected to drought treatment alone (Fig 4).

**Fig 4:** Foliar glycinebetaine (GB) spray on the leaves of pear seedlings under drought tension at the endogenous GB stage. The foliage was sprayed on pear plants with a GB solution of 0 (Drought), 100 (GB 100 + drought) or 500 mg L−1 (GB 500 + drought). Well-watered plants with the same volume of water were also sprayed. On the third and sixth days of the GB foliar spray (or water retention), the soil water levels and leaf water capacity culminated in both the "dryness" and the "GB + drought" classes feeling mild and severe drought tension. Important discrepancies are shown between asterisks and well-watered plants (* *P* < 0.05, ** *P* < 0.01, Student′s *t*-test). Six replicates of the data are shown as the mean ± SD.

### The effects of GB application at the dehydrated detached block level of MDA

We also examined MDA levels in the dehydrated detached leaves to further study the physiological mechanisms of GB involved in drought tolerance. Use of the GB infiltration technique at various concentrations on unwrought leaves revealed that dehydrated GB-nonwrought leaves (0 mg L^−1^ GB, Fig 5A) exhibited significantly higher levels of MDA than nonwrought leaves (0.0 mg L^−1^ GB, Fig 5A). The dehydration-induced MDA increased was dramatically suppressed in a dose-dependent manner by GB application (Fig 5A). In leaves pretreated with 50 mg L^−1^ GB, no significant change was observed at the MDA level. In dehydrated leaves, MDA levels decreased significantly by approximately 20 to 30% compared to dehydrated leaves that were not treated with GB (Fig 5A); however, at 100–1000 mg L^−1^ pretreatment, a phytotoxicity of 5,000 mg L^–1^ GB (not shown) was achieved.

**Fig 5:** Glycinebetaine (GB) therapy’s dose-(A) and time-dependent (B) impact on the severed pear leaves and MDA material. Detached pear leaves were infiltrated with GB solution at varying concentrations for 10 min and permitted to lose water in natural fresh weight (A) or for a separate period (B) through up to 15% evaporation. MDA content was calculated as defined in the Materials and methods section. A was used as a control for nondehydrated leaves that had not been treated with GB (0’). Substantial variations in regulation (0’) were observed (** *P* < 0.01, Student′s *t*-test). Three replicates are shown as means ± SD.

Moreover, using the infiltration technique for testing the timing of GB-inducing effects, application of 500 mg L^−1^ GB on the detached leaves revealed that MDA levels in the GB-treated and -untreated leaves did not change beyond the first 60 min following removal of the leaves from the solution (Fig 5B). In the GB untreated leaves, with incremental wastage, the GB-treated dehydrated leaves displayed a steady increase in MDA content after 60 min of gradually increasing levels (Fig 5B). When the leaves lost approximately 20% of their initial fresh weight at 180 min, we noticed that the MDA amount of dehydrated GB-purposed leaves was slightly below (36%) that of dehydrated GB-purpose leaves (Fig 5B). These results indicate the time-course-dependent inhibitory effects of GB on MDA production.

### Results of GB implementation and SOD activity in dehydrated disconnected leaves

Drought-induced SOD activity was substantially improved in a dose- and time-dependent manner by GB pretreatment of the disconnected leaves (Fig 6A and 6B). Untreated GB leaves exhibited dramatically improved SOD activity compared to nondehydrated GB leaves (0 mg L^–1^ GB, Fig 6A). Additionally, increased SOD levels were observed in 50–1000 mg L^−1^ GB-treated dehydrated leaves, but no substantial difference was noted between the 50 mg L^−1^ GB dehydrated leaves and the GB-untreated dehydrated leaves (Fig 6A). Dehydration with 100 and 1000 mg L^−1^ GB caused substantially greater SOD activity than the untreated GB dehydrated leaves (Fig 6A) compared to 33 and 54% SOD activity.

**Fig 6:** Glycinebetaine (GB) treatment affects SOD activity in severed pear leaves in a dose- (A) and time-dependent manner (B). Detached pear leaves were treated with varying amounts with a GB solution for 10 min, and their water was then spontaneously lost through up to 15% evaporation or for a different duration (B) of the initial fresh weight (A). As described in the Materials and methods section, SOD activity was determined. In A, nondehydrated, non-GB-treated leaves were used as controls (0’). Important contrast is shown by the asterisks compared to the controls (0’) (** *P* < 0.01, Student′s *t*-test). Three replicates are shown as means ± SD.

Furthermore, no improvement in SOD behavior was observed in either GB-treated or nontreated leaves within the first 60 min after the leaves were removed from the solution (Fig 6B). SOD activity levels quickly increased after 60 min, as the activity of SOD steadily increased over time in uncured GB leaves in dehydrated GB-treated leaves (Fig 6B). At 180 min, the dehydrated leaves treated with GB were 42% more active than GB untreated leaves (Fig 6B), and SOD activity was 42% greater.

## Discussion

To mitigate the adverse impact of drought, plants have accumulated in a number of processes, such as cellular osmotic modification, ROS detoxification, membrane integrity defense, and protein and enzyme stabilization [32, 41, 69]. However, in different plants exposed to environmental tension, such as dryness, the accumulation of endogenous GBs is inadequate to control these processes [70]. Exogenous treatment with GB can therefore help decrease the adverse effects of environmental stress, particularly in many GB-accumulating plants, such as sun flowers [29], duckweed [66], pea [68] and wheat [67, 68, 71], and endogenous GB levels are improved in response to exogenous GB treatment. Similarly, this study indicates that application of foliar GB increases the rate of accumulation of endogenous GB in the pear floor (Fig 4).

Drought tension causes numerous adverse effects induced by ROS in plants [72]. During different metabolic cycles, ROS development is normal [73]. However, ROS development, particularly in the case of O_2_·^−^ and H_2_O_2_, increases intracellularly when plants are exposed to drought stress as a typical response to environmental stress in almost all plant species [10, 65, 74, 75]. The current research shows a substantial rise in the output of both O_2_·^−^ and H_2_O_2_ over the well-watered control, which constantly and steadily increased as the stress level increased. (Fig 1), indicating that there was an imbalance in ROS production in dry-stressed pear leaves. Drought-tolerant multiplant cultivars include rice [65] and alfalfa [76]. Compared to vulnerable dry crop crops, lower levels of O_2_·^−^ and H_2_O_2_ are correlated with reduced development of ROS resistance [65].

The stress-induced increase in both O_2_·^−^ and H_2_O_2_ in pear leaves was greatly decreased by GB application (Fig 1), whereas the GB-mediated decrease in ROS output coincided with increased endogenous GB levels (Fig 4). Previous reports have revealed the efficacy of GB in attenuating abiotic stress-induced ROS [77–79].

Excessive ROS development is likely to cause rapid cellular damage, including lipid peroxidation of cell membranes, by causing a chain reaction [80]. MDA [66, 81] is a typical product of lipid peroxidation used to indicate the level of oxidative stress on plant cells. Stressed pear leaves exhibited higher MDA levels than well-watered controls (Fig 2A), in accordance with enhanced O_2_·^−^ and H_2_O_2_ output, which was followed by significantly elevated EL levels (Fig 2B), explaining the loss of the physical permeability of the cell membranes. Exogenous application of GB significantly decreased both MDA and EL concentrations in dry pear leaves (Fig 2), indicating that GB-treated stressed pear leaves experienced reduced oxidative damage. The decrease in the MDA content and EL in response to GB in stressed pear leaves is proof of the major improvement in the adverse effects of drought on membrane integrity and stabilization of pear leaves by exogenous GB application.

Plants have also evolved ROS-induced repair and protection mechanisms. These mechanisms include antioxidant enzymes, such as SOD, POD and CAT [66]. SOD constitutes the first response against ROS and catalyzes dismutation using a broad variety of antioxidant enzymes from O_2_·^−^ to O_2_ and H_2_O_2_ [82], and POD and CAT have the most significant effects [35]. The current research indicates a large increase in SOD activity in drought-stressed leaves (Fig 3A). Elevated SOD activity has also been linked to stress resistance in plants, while conflicting findings were observed in barley in Kubi [74] under water deficiency conditions [65, 83–87].

Exogenous treatment with GB in maize [35] and rice [78] under drought stress conditions has been previously documented to improve SOD activity. However, exogenous GB therapy for salt-stressed rice seedlings has also been found to decrease SOD activity [49]. These contrasting findings may be attributed to species-specific and cultivar-specific efficacies of GB application for the regulation of antioxidant enzyme activities [71]. This research consistently shows that the whole pear plant and detached leaf studies exhibited greatly improved SOD activity in drought-stressed leaves in response to exogenous GB application (Figs 3A and 6). In addition, the increase in SOD activity induced by GB was associated with increased concentrations of endogenous GB and reduced O_2_·^−^ levels (Figs 1A, 3A and 4). This evidence supports the contribution of GB to the detoxification of O_2_·^−^ radicals by improving SOD activity in pear leaves under conditions of drought stress.

In terms of POD behavior, we observed a related pattern (Fig 3B). Dry pear plants without GB administration displayed considerably increased POD activity relative to the well-watered controls after 3 d, whereas PODs from dry-powered plants without GB application contributed to even greater POD activity levels in drought-stressed leaves compared to drought-induced PODs without GB administration (Fig 3B). We also found that the rise in activity from GB-induced POD was associated with increased endogenous levels of GB and was followed by a reduction in GB level from H_2_O_2_ at the same time (Figs 1B, 3B and 4), indicating that GB possibly contributes to the detoxification of H_2_O_2_ by increasing POD activity in pear leaves under conditions of drought stress.

CAT is found in higher plant peroxisomes and leads to H_2_O_2_ decomposition [82]. CAT plays an essential function in guarding against oxidative stress amid its minimal localization [82]. In the current research, however, only minor changes in CAT activity were found in the leaves of pear plants exposed to dry stress (Fig 3C). Foliar application of GB considerably elevated CAT activity in drought-stressed leaves relative to well-watered leaves, but this increase was not substantial (Fig 3C), indicating that in drought-stressed pear leaves, CAT might be a less efficient H_2_O_2_ scavenger.

## Conclusions

In conclusion, exogenous application of foliar GB decreased oxidative harm in pears under drought stress by reducing the aggregation of ROS, such as O_2_·^−^ and H_2_O_2_, in cells. In the sense of ROS scavenging, GB applications played more essential roles in improving SOD, CAT and POD activities. In addition, GB application greatly decreased the adverse effects of dry stress on membrane integrity and resilience in drought-stressed pear leaves by reducing both MDA and EL levels. Our results suggest that the use of exogenous GB should be considered in studies that are involved in designing strategies for the control of drought tolerances. Our study shows some of the processes underpinning the mechanism for how GB treatment increases drought resistance of a woody pear species, which can be used for successful control of drought stresses in pear farming.
